# miR-494-3p Promotes Erastin-Induced Ferroptosis by Targeting REST to Activate the Interplay between SP1 and ACSL4 in Parkinson's Disease

**DOI:** 10.1155/2022/7671324

**Published:** 2022-07-29

**Authors:** Jianjun Ma, Xiaohuan Li, Yongyan Fan, Dawei Yang, Qi Gu, Dongsheng Li, Siyuan Chen, Shaopu Wu, Jinhua Zheng, Hongqi Yang, Xue Li

**Affiliations:** ^1^Department of Neurology, Henan Provincial People's Hospital, Zhengzhou, Henan 450003, China; ^2^Department of Neurology, Zhengzhou University People's Hospital, Zhengzhou, Henan 450003, China; ^3^Department of Neurology, Henan University People's Hospital, Zhengzhou, Henan 450003, China

## Abstract

**Background:**

Ferroptosis is a type of iron-dependent programmed cell death. Ferroptosis has been shown to be a significant factor for the pathogenesis of Parkinson's disease (PD). However, the mechanism involved in ferroptosis has not been fully elucidated in PD.

**Methods:**

Repressor element-1 silencing transcription factor (REST) and specificity protein 1 (SP1) expressions were monitored by qRT-PCR. Cell viability, reactive oxygen species (ROS), and mitochondrial injury were validated by CCK-8, flow cytometry, and transmission electron microscope. The levels of neurons-related proteins and ferroptosis-associated proteins were identified by western blot and immunofluorescence assays. The interaction between miR-494-3p and REST or SP1 and ACSL4 was analyzed by luciferase, chromatin immunoprecipitation, or EMSA assay.

**Results:**

Erastin could dose-dependently induce neuron injury and ferroptosis of LUHMES cells. miR-494-3p overexpression induced ROS production, mitochondrial damage, ferroptosis, and neuron injury in erastin-induced LUHMES cells. Likewise, miR-494-3p inhibition had the opposite effects. We also showed that REST was a target gene of miR-494-3p and could repress erastin-induced ferroptosis, neuron injury, ROS, and mitochondrial injury via SP1 in LUHMES cells. Moreover, we demonstrated that SP1 could interact with ACSL4. We also confirmed that miR-494-3p could aggravate the pathological changes of substantia nigra and corpus striatum in the MPTP-induced PD mouse model.

**Conclusion:**

miR-494-3p significantly promotes ferroptosis by regulating the REST/SP1/ACSL4 axis in PD. Thus, our results open potential therapeutic targets for PD.

## 1. Introduction

Parkinson's disease (PD) is the second most common neurodegenerative disease after Alzheimer's. The primary pathological features of PD are the degeneration and loss of dopaminergic neurons in substantia nigra pars compacta of the midbrain [1–3]. Studies manifested that PD can cause static tremor, muscle rigidity, sleep disorders, bradykinesia, abnormal attitudinal reflexes, sensory disorders, autonomic nervous dysfunction, and other clinical manifestations [4, 5]. It has been reported that many factors are involved in the occurrence of PD, including the environment, genetics, aging, oxidative stress, inflammation, mitochondrial dysfunction, lack of neurotrophic factors, and abnormal accumulation of iron [6–8]. Meanwhile, various cell death modes, including apoptosis, autophagy, and necrosis, also participate in the pathological process of PD [9, 10]. However, the pathogenesis of PD is still not fully understood in the existing studies.

Ferroptosis is a new type of cell death caused by iron-dependent oxidative damage, which is different from apoptosis, necrosis, and autophagy in aspects of morphology, biochemistry, and genetics [11]. As a mode of iron-dependent cell death, iron has a significant effect on ferroptosis [12]. Neuroimaging examination and autopsy pathology report of PD patients confirmed a large amount of iron deposition in the substantia nigra and increased iron content in the remaining dopaminergic neurons. Iron selectively aggregates in the substantia nigra in early PD patients, suggesting that iron can be served as a biomarker and imaging indicator to reflect the progression of PD [13]. Recent researches also verified that ferroptosis could facilitate PD progression [14, 15]. However, the mechanism of ferroptosis involvement in the degeneration of dopaminergic neurons in PD substantia nigra is still unclear. Therefore, a better understanding of the pathogenesis of ferroptosis in PD will aid in providing new ideas for PD therapy.

MicroRNAs (miRNAs) are a class of cellular endogenous, highly conserved, noncoding small RNA molecules, approximately 21-25 nucleotides in length [16]. The main function of miRNAs is to regulate gene expression at the transcriptional level to exert physiological functions [17]. It has been reported that miRNAs can participate in cell proliferation, differentiation, apoptosis, inflammatory response, autophagy, and other biological characteristics [18]. And miRNAs are also associated with neurodegenerative diseases, including PD [19, 20]. Meanwhile, miRNAs, such as miR-137, miR-424-5p, and miR-30-5p, were proven to be relevant to ferroptosis [21]. Moreover, the latest study showed that miR-494-3p could induce PD progression by SIRT3 [22], and pramipexole could prevent neurotoxicity by miR-494-3p in PD [23]. Through literature screening, we also found that miR-494-3p is associated with multiple diseases, including myocardial infarction [24], lung cancer [25], and hepatocellular carcinoma [26]. while the function and mechanism of miR-494-3p in ferroptosis-mediated PD are still broadly unknown.

In the current study, we verified the potential function and mechanism of miR-494-3p in PD through *in vivo* and *in vitro* experiments, especially the regulation of ferroptosis, which may provide a novel target for PD treatment.

## 2. Materials and Methods

### 2.1. Cell Treatment

To establish the ferroptosis cell model, different concentrations (0, 0.25, 0.5, 1, 2, and 4 *μ*M) of erastin (Tocris, USA) were used to stimulate the LUHMES for 24 hours [27, 28]. Negative control (NC), miR-494-3p mimics, and miR-494-3p inhibitor were purchased from GenePharma (Suzhou, China). Empty vector, REST-overexpressed plasmids, SP1-overexpressed plasmids, REST shRNAs (sh-REST), and sh-NC were acquired from Hanbio Biotechnology (China). In 6-well plates, LUHMES cells (5 × 10^4^ cells/well) were transfected with these oligodeoxynucleotides or overexpressed plasmids using Lipofectamine 3000 (Invitrogen) for 48 hours based on the specification. 100 nM ferroptosis inhibitor (ferrostatin-1, Selleck, USA) or mithramycin was added to the erastin-stimulated LUHMES cells for 1 hour [29].

### 2.2. Animal

Healthy C57BL/6 male mice (weight 20 ± 1 g) were purchased from the Henan Experimental Animal Center and kept in the Henan Experimental Animal Center with temperature (24°C ± 2°C), humidity (55% ± 5%), and 12 hours light/12 hours darkness and sterile water. The Ethics Committee of Henan University People's Hospital has approved the animal experiment (No. 2019-76). PD mouse model was established by intraperitoneal injection of 30 mg/kg 1-methyl-4-phenyl-1,2,3,6-tetrahydropyridine (MPTP; Sigma, Cat. no. MO896) for 7 days [30]. Then, PD model mice were randomly divided into 6 groups: sham (*n* = 8, mice were intraperitoneally injected with 30 mg/kg normal saline for 7 days), MPTP (*n* = 8, mice were intraperitoneally injected with 30 mg/kg MPTP for 7 days), MPTP+NC (*n* = 8, a stereotactic catheter was implanted into the right lateral ventricle of MPTP-treated mice through surgery, and NC was injected through the catheter for 5 days), MPTP+miR-494-3p antagomir (*n* = 8, 5 *μ*L of saline with 20 nmol/L miR-494-3p antagomirs was injected through the catheter for 5 days in the MPTP-treated mice), MPTP+miR-494-3p agomir (*n* = 8, 5 *μ*L of saline with 20 nmol/L miR-494-3p agomir was injected through the catheter for 5 days in the MPTP-treated mice) [31, 32], and MPTP+ferrostatin-1 (*n* = 8, mice were injected with 2.5 mM ferrostatin-1 via ventricle 1 day before the MPTP intoxication) groups [33]. The mice were sacrificed through cervical dislocation at the end of the experiment, the brain was removed, and substantia nigra and corpus striatum were isolated and stored at −80°C.

### 2.3. Immunofluorescence Assay

LUHMES cells in each group were grown on coverslips, fixed with 4% paraformaldehyde for 20 min, and permeated using 0.5% Triton X-100 (Sigma-Aldrich) for 20 min. For the tissue sections, the slices of substantia nigra and corpus striatum were dewaxed with xylene, treated with gradient alcohol, and washed with PBS. Subsequently, the slices were subjected to antigen repair by microwave with citrate. After cooling to room temperature, the slices were treated with 3.3% H_2_O_2_ at 37°C for 20 min. After washing and blocking, the samples were incubated with anti-ACSL4 (1 : 50 dilution, Abcam, ab227256) and anti-TH (1 : 50 dilution, Abcam, ab137721) overnight at 4°C, then with the corresponding secondary antibody (Abcam) for 1 hour. The nuclei were stained using 10 g/mL DAPI, and the results were immediately photographed under a fluorescence microscope. For details of other experimental methods, please refer to the supplementary materials (available here).

### 2.4. Statistical Analysis

All data were expressed as mean ± SD from three independent replicates. The data was calculated using SPSS software 23.0 (SPSS Inc., Chicago, IL, USA) with a one-way analysis of variance (ANOVA) followed by post hoc Newman–Keuls multiple comparisons. *P* < 0.05 was considered statistically significant.

## 3. Results

### 3.1. Different Concentrations of Erastin Induce Ferroptosis and Upregulate miR-494-3p in the LUHMES Cells

To establish the ferroptosis cell model, we applied different concentrations of erastin (0, 0.25, 0.5, 1, 2, and 4 *μ*M) to stimulate LUHMES cells for 24 hours. qRT-PCR results showed that the level of miR-494-3p was gradually elevated in the erastin treatment compared to the control groups. We found a dose-dependent relationship between the upregulation of miR-494-3p and the increase of erastin concentration (*P* < 0.05, *P* < 0.001, Figure 1(a)). Meanwhile, CCK-8 data uncovered that the proliferation activity of LUHMES cells gradually decreased with the increase in erastin concentration (*P* < 0.01, *P* < 0.001, Figure 1(b)). Moreover, the western blots demonstrated that erastin induction markedly downregulated TH, NSE, and GPX4 and upregulated ACSL4 in LUHMES cells (*P* < 0.05, *P* < 0.01, *P* < 0.001, respectively, Figures 1(c) and 1(d)). Thus, the ferroptosis cell model was successfully built through erastin stimulation, and 4 *μ*M erastin had the strongest inducing effect.

### 3.2. Inhibition of miR-494-3p Suppresses Ferroptosis, Neuron Injury, and Reactive Oxygen Species (ROS) Production and Induces Viability in Erastin-Induced LUHMES Cells

Subsequently, we treated erastin-stimulated LUHMES cells with miR-494-3p inhibitor, miR-494-3p mimics, or ferroptosis inhibitor (ferrostatin-1). The qRT-PCR data revealed that relative to the control LUHMES group, the expression level of miR-494-3p was significantly increased in the erastin-stimulated LUHMES cells (*P* < 0.01). Meanwhile, the increase in miR-494-3p level was substantially reduced by miR-494-3p inhibitor and ferrostatin-1 in the erastin-stimulated LUHMES group (*P* < 0.001, Figure 2(a)). Furthermore, CCK-8 data showed that erastin memorably inhibited the proliferation of LUHMES cells, while this inhibition was weakened by miR-494-3p inhibitor and ferrostatin-1 (*P* < 0.05, *P* < 0.01, and *P* < 0.001, Figure 2(b)). And our results discovered that erastin dramatically enhanced ROS activity in LUHMES cells, while miR-494-3p inhibitor and ferrostatin-1 partially rescued the enhancement of ROS activity in erastin-stimulated LUHMES cells (*P* < 0.01, *P* < 0.001, Figures 2(c) and 2(d)). Furthermore, transmission electron microscopy (TEM) results revealed that in the control group, the mitochondrial structure in the LUHMES cells was complete with many mitochondria and visible cristae. In contrast, in the erastin group, the mitochondria had local edema, disordered cristae, and vacuolar degeneration; in the erastin+miR-494-3p inhibitor and erastin+ferrostatin-1 groups, mitochondria were abundant and normal in shape, and cristae are visible; in erastin+miR-494-3p mimics, the degree of mitochondrial injury was more severe than that in the erastin group (Figure 2(e)). Moreover, western blotting data showed that neuron injury-related proteins (TH and NSE) and GPX4 were significantly downregulated, and ACSL4 was strikingly upregulated in erastin-stimulated LUHMES cells compared to that in controls. Meanwhile, the above effect was markedly reversed by miR-494-3p inhibitor or ferrostatin-1 (*P* < 0.01, *P* < 0.001, Figure 2(f)).

### 3.3. REST Is a Target Gene of miR-494-3p

The underlying mechanism was further identified by which miR-494-3p inhibition prevents ferroptosis, thus affecting the progression of PD. qRT-PCR and western blot results showed that miR-494-3p inhibition or ferrostatin-1 dramatically upregulated REST, and miR-494-3p overexpression significantly downregulated REST in erastin-induced LUHMES cells (*P* < 0.05, *P* < 0.001, Figures 2(g) and 2(h)). Moreover, through bioinformatics, we discovered two latent binding sites between miR-494-3p and REST, indicating that REST might be a target gene of miR-494-3p. Then, we constructed the plasmids of WT-REST and Mut-REST and conducted a dual-luciferase reporter assay with miR-494-3p mimics. The luciferase activity of WT-REST was notably attenuated after the cotransfection of miR-494-3p mimics. However, the luciferase activity of Mut-REST did not change, which suggested that REST is a direct target of miR-494-3p (*P* < 0.05, Figure 2(i)).

### 3.4. REST Inhibits Ferroptosis, Neuron Injury, and ROS Production and Accelerates Viability in Erastin-Induced LUHMES Cells

Next, we further validated the effects of REST alteration on the related functions of erastin-induced LUHMES cells. The erastin-induced LUHMES cells were transfected with REST-overexpressed plasmid or sh-REST. qRT-PCR analysis validated that REST overexpression increased REST expression, and REST knockdown decreased REST expression in erastin-induced LUHMES cells, indicating the successful transfection of REST-overexpressed plasmid or sh-REST (*P* < 0.01, *P* < 0.001, Figure 3(a)). CCK-8 data showed that overexpression of REST dramatically enhanced, and knockdown of REST significantly prevented the viability of erastin-induced LUHMES cells (*P* < 0.05, *P* < 0.01, *P* < 0.001, Figure 3(b)). Flow cytometer data showed that overexpression and knockdown of REST significantly reduced and increased the ROS levels, respectively, in erastin-induced LUHMES cells (*P* < 0.01, *P* < 0.001, Figures 3(c) and 3(d)). Furthermore, TEM images also uncovered that overexpression of REST observably alleviated mitochondrial injury, and knockdown of REST memorably aggravated the mitochondrial injury in erastin-induced LUHMES cells (Figure 3(f)). Moreover, western blotting data highlighted that overexpression of REST upregulated REST, TH, NSE, and GPX4 and downregulated ACSL4 in erastin-induced LUHMES cells. Knockdown of REST exerted the opposite effect of overexpression-mediated expression change of these proteins (*P* < 0.05, *P* < 0.01, *P* < 0.001, Figure 3(f)).

### 3.5. REST Attenuates the Effect of miR-494-3p on Viability, ROS, Ferroptosis, and Neuron Injury in Erastin-Induced LUHMES Cells

Subsequently, we conducted the rescue experiments to investigate whether REST can be involved in blocking PD mediated by miR-494-3p downregulation by inhibiting ferroptosis. Erastin-stimulated LUHMES cells were first cotransfected with miR-494-3p inhibitor and sh-REST or REST-overexpressed plasmid and miR-494-3p mimics. The qRT-PCR data showed that knockdown of REST upregulated miR-494-3p mediated by miR-494-3p inhibitor, whereas overexpression of REST significantly downregulated miR-494-3p mediated by miR-494-3p mimics in erastin-induced LUHMES cells (*P* < 0.05, *P* < 0.01, Figure 4(a)). And we also showed that knockdown of REST significantly reduced REST expression mediated by miR-494-3p inhibitor, and overexpression of REST markedly raised REST expression mediated by miR-494-3p mimics in erastin-induced LUHMES cells (*P* < 0.01, Figure 4(b)). Likewise, CCK-8 data demonstrated that knockdown of REST dramatically attenuated viability mediated by miR-494-3p inhibitor, whereas overexpression of REST remarkably enhanced viability mediated by miR-494-3p mimics in erastin-induced LUHMES cells (*P* < 0.05, *P* < 0.01, Figure 4(c)). The flow cytometry results disclosed that REST knockdown significantly elevated ROS level mediated by miR-494-3p inhibitor and REST overexpression significantly lowered ROS level mediated by miR-494-3p mimics in erastin-induced LUHMES (*P* < 0.05, Figure 4(d)). Meanwhile, TEM images showed that REST knockdown markedly induced mitochondrial injury mediated by miR-494-3p inhibitor, and REST overexpression prevented mitochondrial damage mediated by miR-494-3p mimics in erastin-induced LUHMES cells (Figure 4(e)). Meanwhile, immunofluorescence assay also uncovered that REST silencing could upregulate ACSL4 and downregulated TH mediated by miR-494-3p inhibitor and downregulate ACSL4 and upregulated TH mediated by miR-494-3p mimics in erastin-induced LUHMES cells (Figures 4(f) and 4(g)). Furthermore, we proved that REST silencing downregulated REST, TH, NSE, and GPX4 and upregulated ACSL4, which were mediated by miR-494-3p inhibitor, and REST overexpression upregulated REST, TH, NSE, and GPX4 and downregulated ACSL4, which were mediated by miR-494-3p mimics in erastin-induced LUHMES (*P* < 0.05, *P* < 0.01, *P* < 0.001, Figure 4(h)).

### 3.6. SP1 Reverses the Roles of REST on Viability, ROS, Ferroptosis, and Neuron Injury in Erastin-Induced LUHMES Cells

Moreover, we further verified whether SP1 could participate in blocking the PD progression mediated by REST by inhibiting ferroptosis and whether SP1 also can participate in the inhibition effect of REST on PD progression. Erastin-stimulated LUHMES cells were coprocessed with REST and SP1 overexpressing plasmids or REST shRNAs (sh-REST) and mithramycin. The results unveiled that overexpression of REST significantly reduced SP1 expression and transcription factor activity in erastin-stimulated LUHMES cells; this expression and transcription factor activity of SP1 mediated by REST overexpression could be notably potentiated by SP1 overexpression. Meanwhile, silencing of REST significantly elevated SP1 expression and transcription factor activity in erastin-stimulated LUHMES cells. This elevation mediated by REST silencing could be observably attenuated by mithramycin (*P* < 0.05, *P* < 0.01, *P* < 0.001, Figures 5(a) and 5(b)). Then, we utilized an SP1 transcription factor assay to identify SP1 activity in REST overexpressed or silenced LUHMES after erastin induction. The data revealed that overexpression of REST markedly lowered SP1 activity, and knockdown of REST prominently lowered SP1 activity in erastin-induced LUHMES (*P* < 0.001, Figure 5(c)). Subsequently, we found that overexpression of REST enhanced the viability of erastin-stimulated LUHMES cells, while this enhancement was remarkably weakened by SP1 overexpression. On the other hand, silencing of REST markedly reduced the viability of erastin-stimulated LUHMES cells, while this reduction was significantly reversed by mithramycin (Figure 5(d)). Furthermore, we found that overexpression of REST dramatically diminished ROS activity of erastin-stimulated LUHMES cells, while this reduction was weakened by SP1 overexpression. Silencing of REST markedly improved ROS activity of erastin-stimulated LUHMES cells, while this improvement was markedly reversed by mithramycin (*P* < 0.01, *P* < 0.001, Figure 5(e)). And the TEM data indicated that REST overexpression prominently mitigated mitochondrial injury of erastin-stimulated LUHMES cells, while this mitigation was weakened by SP1 overexpression. REST silencing memorably accelerated mitochondrial injury of erastin-stimulated LUHMES, while mithramycin significantly reversed this acceleration (Figure 5(f)). Besides, immunofluorescence results demonstrated that SP1 overexpression could reverse the downregulation of ACSL4 and upregulation of TH, mediated by REST overexpression. Similarly, mithramycin also could reverse the upregulation of ACSL4 and downregulation of TH, mediated by REST silencing in erastin-stimulated LUHMES cells (Figures 5(g) and 5(h)). The results also revealed that overexpression of REST downregulated SP1 and ACSL4 and upregulated TH, NSE, and GPX4, which was reversed by SP1 overexpression. Knockdown of REST upregulated SP1 and ACSL4 and downregulated TH, NSE, and GPX4, which was also significantly reversed by mithramycin (*P* < 0.05, *P* < 0.01, *P* < 0.001, Figure 5(i)).

### 3.7. SP1 Can Target ACSL4

The specific mechanism was further understood by which SP1 influences ferroptosis. Bioinformatics analysis suggested that ACSL4 might be the downstream target gene of SP1. We also explored the binding sites between SP1 and ACSL4 (Figure 6(a)). Then, dual-luciferase reporter assay showed that SP1 significantly enhanced the promoter activity of ACSL4 (two binding sites) relative to the respective wild-type ACSL4 promoter, suggesting that SP1 could target ACSL4 (*P* < 0.001, Figures 6(b) and 6(c)). A chromatin preparation was precipitated with anti-SP1, and the immunoprecipitated DNA fragments were amplified with the primers, including the ACSL4 binding site. Chromatin immunoprecipitation (CHIP) results suggested that DNA fraction was immunoprecipitated with the anti-SP1 while none with the IgG (negative control), indicating SP1 could bind to ACSL4 (*P* < 0.001, Figure 6(d)). Likewise, electrophoretic mobility shift (EMSA) results also showed that SP1 and ACSL4 could interact directly (Figure 6(e)).

### 3.8. miR-494-3p Aggravates Pathological Changes, Upregulates ACSL4, and Downregulates TH in the Substantia Nigra and Corpus Striatum of the MPTP-Induced PD Mouse Model

Furthermore, we established a PD mouse model through MPTP induction and examined the influence of miR-494-3p and ferrostatin-1 on the pathological changes and ACSL4 and TH expressions in substantia nigra and corpus striatum. The qRT-PCR data showed that relative to sham mice, miR-494-3p was upregulated, and REST was downregulated in the MPTP-induced PD model mice. Inhibition of miR-494-3p or ferrostatin-1 downregulated miR-494-3p and upregulated REST. Further, overexpression of miR-494-3p upregulated miR-494-3p and downregulated REST in MPTP-induced PD model mice, suggesting the successful treatment of the PD mouse model (*P* < 0.05, *P* < 0.01, Figures 7(a) and 7(b)). Then, hematoxylin and eosin (H&E) staining demonstrated that the number of neurons in the sham group was relatively dense and orderly, and the stroma was clear. However, in the PD model group, the neurons were disordered, the number of neurons was reduced, the contour of the cell body was blurred, the cytoplasm was swollen, and some vacuolar degeneration or shrinkage necrosis was observed. These conditions improved in the miR-494-3p antagomir and ferrostatin-1 treatment groups and worsened in the miR-494-3p agomir group (Figure 7(c)). Immunofluorescence results then showed that ACSL4 expression was elevated in the substantia nigra and corpus striatum of the MPTP-induced PD mice compared to sham mice. Inhibiting miR-494-3p or ferrostatin-1 dramatically downregulated ACSL4, and overexpression of miR-494-3p observably upregulated ACSL4 in the MPTP-induced PD model mice (Figure 7(d)). Similarly, immunohistochemistry results showed that TH expression was reduced in the MPTP-induced PD model mice's substantia nigra and corpus striatum relative to that in the sham mice. Inhibition of miR-494-3p or ferrostatin-1 dramatically increased TH expression, and overexpression of miR-494-3p signally decreased TH expression in MPTP-induced PD model mice (Figure 7(e)).

## 4. Discussion

PD is one of the most common neurodegenerative diseases of the central nervous system [2]. However, the etiology and pathogenesis of PD are still broadly unknown. Recent studies demonstrated that the midbrain of PD patients is characterized by high iron content, low glutathione, and increased lipid peroxidation, suggesting that the pathogenesis of PD is relevant to ferroptosis [15, 34]. Ferroptosis is a newly discovered form of cell death, which can be induced by a variety of chemical and biological factors [35]. It is mainly characterized by iron-dependent lipid peroxidation leading to cell death. Metabolism of iron, lipid, and amino acid is the main pathway to regulate ferroptosis, which can be antagonized by GPX4 and FSP1 [36]. Studies also indicated that ferroptosis could be rescued by small molecules, such as desferrioxamine and ferrostatin-1 [37]. Besides, ferroptosis is a gene-regulated form of cell death. In different diseases, ferroptosis can be regulated by multiple regulatory molecules, such as GPX4, ACSL4, SLC7A11, and TFR1 [38, 39]. Several ferroptosis inhibitors have demonstrated a strong ability to alleviate PD [40]. Therefore, further studying the primary regulatory mechanism of ferroptosis in PD might provide an underlying target for PD treatment.

Erastin is a small tumor growth suppressor molecule that selectively targets oncogene RAS. Erastin mainly prevents cystine uptake through the cystine/glutamate transport system, avoids the protection of antioxidants, and eventually leads to iron-dependent and lipid ROS-dependent oxidation death, called ferroptosis [41]. This study also established the ferroptosis PD cell model through erastin induction in LUHMES cells based on previous research [42]. We showed that erastin, especially with 4 *μ*M, suppresses proliferation and accelerates ferroptosis in LUHMES cells, indicating that the ferroptosis PD cell model was successfully established by erastin stimulation. Epidemiological investigation testified that occupational exposures to heavy metals, pesticides, herbicides, and other environmental factors might be a risk factor for PD [43]. Earlier studies also discovered that the injection of 1-methyl-4-phenyl-1,2,3,6-tetrahydropyridine (MPTP) could result in symptoms like PD [44]. As previously reported, iron was significantly increased in the substantia nigra of MPTP-induced PD mice and the remaining dopaminergic neurons [45]. An iron-chelating agent can protect the neurotoxic model induced by MPP^+^ [46]. The specific iron deposition in the substantia nigra is a crucial factor in the damage of dopaminergic neurons in PD [8]. We also chose MPTP to generate the chronic PD mouse model in this study. We showed the pathological structure unfavorably changes in the substantia nigra and corpus striatum of PD mice, suggesting that the PD mouse model was successfully generated.

Besides, our results uncovered that miR-494-3p was dramatically upregulated in erastin-induced LUHMES and MPTP-induced PD mice, suggesting that miR-494-3p might participate in the PD process. Downregulation of miR-494-3p could attenuate neurotoxicity of SK-N-SH and CHP 212 cells, suggesting that inhibition of miR-494-3p might be a latent method of PD therapy [23]. In our study, we also showed that inhibition of miR-494-3p could weaken neuron injury and enhance the viability of erastin-induced LUHMES, suggesting the protective effect of miR-494-3p inhibition on PD model cells induced by erastin. We also demonstrated that inhibition of miR-494-3p, consistent with ferrostatin-1, could suppress ferroptosis and ROS production in PD model cells induced by erastin. Moreover, we found that inhibition of miR-494-3p could improve pathological changes and ferroptosis in substantia nigra and corpus striatum of MPTP-induced PD model mice. Thus, our results indicate that inhibition of miR-494-3p might relieve PD by inhibiting ferroptosis.

As a DNA zinc-finger binding protein, REST can induce histone deacetylation and transcriptional inhibition of target genes by binding with neuron-restrictive silencer element (NRSE) [47]. REST, as a key negative transcriptional regulator in the nervous system, is widely involved in neuronal growth and differentiation, axon growth, vesicle transport and release, and ion conduction [47]. Therefore, REST plays a role in regulating various aspects of nerve function, such as cell differentiation, nerve regeneration, nerve protection, and cognitive function [48]. Researchers also discovered that REST plays multiple roles in different neurological diseases, especially PD [49]. REST also has a protective effect on numerous stress stimulations and can maintain neuronal activity through antioxidative stress [50]. In our study, we further confirmed that REST also could inhibit ferroptosis, neuron injury, and ROS production and induce viability of erastin-induced LUHMES cells, suggesting the mitigation role of REST on PD. Moreover, we found that miR-494-3p could bind to REST 3′-UTR through prediction software, suggesting that REST might be the target gene of miR-494-3p. And the results from the dual-luciferase reporter assay verified the same. Meanwhile, the rescue experiments showed that inhibition of miR-494-3p could alleviate PD by targeting REST to inhibit ferroptosis.

SP1 protein is a member of the SP/KLF transcription factor family [51]. SP1 has 4 parts based on its functions: DNA binding region, SP1 active region, Buttonhead (BTD) box, and SP box [51]. Under normal physiological conditions, SP1 is widely expressed in various tissues and organs in the organism and regulates multiple housekeeping genes [52]. Recently, it has been reported that SP1 is associated with oxidative stress and ferroptosis [53]. Meanwhile, SP1 was confirmed to be relevant to PD by several studies. For instance, miR-375 ameliorates dopaminergic neuronal damage by attenuating SP1 to attenuate PD inflammatory response [54]. miR-126-5p targets SP1 to stop PD progression [55]. miR-29c targets SP1 to inhibit PD inflammation and apoptosis [56]. SP1 is involved in MPTP-induced cell damage in PD [57]. In PD models, SP1 inhibition can exert neuroprotective effects [58]. And our results further demonstrated that SP1 also could reverse the roles of REST on viability, ROS, ferroptosis, and neuron injury in erastin-induced LUHMES cells, suggesting that REST also could alleviate PD by reducing SP1 activity. Thus, we uncovered that SP1 is vital in REST-regulated ferroptosis in PD.

Besides, SP1 can interact with other protein molecules to exert a negative regulation on target genes [59]. Study has shown that SP1 can affect the cell cycle, apoptosis, and angiogenesis [60]. Here, we unexpectedly discovered that ACSL4 might be the downstream target gene of SP1 through bioinformatics analysis. Moreover, our data also disclosed that overexpression of REST could downregulate ACSL4 in erastin-induced LUHMES cells. ACSL4 is a crucial enzyme in fatty acid metabolism and a member of the long-chain lipid coenzyme A synthase (ACSL) family [61]. Study has demonstrated that ACSL4 is closely related to animal fat metabolism [62]. In addition, the expression of ACSL4 can affect cancer cell proliferation, migration, invasion, and apoptosis [63, 64]. It has also been found that mutations in the ACSL4 gene cause altered ACSL4 enzyme activity, affecting neurodevelopment [65]. ACSL4 has also been reported to be one of the essential components for triggering cellular ferroptosis through its involvement in the synthesis of membrane phospholipids that are susceptible to oxidation [66–68]. Therefore, we speculated that ACSL4 is likely to be associated with ferroptosis in PD. The role and mechanism of ACSL4 in PD were broadly unknown. In our study, we further certified that ACSL4 is a target gene of SP1. Overall, we showed that inhibition of miR-494-3p could attenuate ferroptosis and PD progression by the REST/SP1/ACSL4 axis.

However, the current study also has limitations that need further study. (i) The specific mechanism between SP1 and REST is still unclear. (ii) The effects of the miR-494-3p/REST/SP1/ACSL4 axis on other related functions of PD, such as oxidative stress, autophagy, apoptosis, and proliferation, remain unanswered. (iii) Although this study verified the role of the miR-494-3p/REST/SP1/ACSL4 axis, we mainly focused on the cellular level, and further verification is also needed in experimental animal studies. (iv) The influence of this signaling pathway on PD patients also needs to be further investigated.

## 5. Conclusion

Our results manifested that inhibition of miR-494-3p could prevent ferroptosis and neuron injury by targeting REST to regulate the SP1/ACSL4 axis in PD. These findings demonstrated that miR-494-3p/REST/SP1/ACSL4 pathway is crucial in regulating PD ferroptosis. Overall, this study revealed that miR-494-3p, REST, SP1, and ACSL4 are in the same signaling axis, and there is a clear upstream and downstream regulatory relationship between them. Therefore, it would be of great clinical application to further explore drugs with functional activity to regulate these four genes and validate whether they can improve PD.

## Figures and Tables

**Figure 1:** Different concentrations of erastin induce ferroptosis and upregulate miR-494-3p in the LUHMES cells. LUHMES cells were stimulated by 0, 0.25, 0.5, 1, 2, and 4 *μ*M erastin for 24 hours. (a) qRT-PCR analysis of miR-494-3p in erastin-stimulated LUHMES cells. (b) Cell proliferation analysis by CCK-8 assay. (c) The levels of TH, NSE, ACSL4, and GPX4 were estimated by western blotting in erastin-stimulated LUHMES cells. (d) Relative protein levels of TH, NSE, ACSL4, and GPX4 based on the western blotting results. Results were representative data from triplicate experiments, and data are means ± SD. ^∗^*P* < 0.05, ^∗∗^*P* < 0.01, and ^∗∗∗^*P* < 0.001.

**Figure 2:** The impact of miR-494-3p on viability, ROS, ferroptosis, neuron injury, and REST in erastin-induced LUHMES cells. Erastin-stimulated LUHMES cells were transfected with miR-494-3p inhibitor, miR-494-3p mimics, or NC or treated with ferroptosis inhibitor (ferrostatin-1). (a) The miR-494-3p level was tested by qRT-PCR assay in each group. (b) Cell proliferation was monitored via CCK-8 assay in the above groups. (c and d) ROS activity was identified via a flow cytometer in each group. (e) TEM images showing mitochondrial morphology in each group. Scale bar = 2 *μ*m. Mitochondria are marked with blue arrows. (f) Western blotting analysis of TH, NSE, ACSL4, and GPX4 in each group. (g and h) qRT-PCR and western blotting analysis of REST. (i) WT and Mut REST 3′-UTR plasmids were constructed and cotransfected with miR-494-3p mimics into cells, and then, the luciferase activity was tested by dual-luciferase reporter assay. Results were representative data from triplicate experiments, and data are means ± SD. ^∗^*P* < 0.05 and ^∗∗∗^*P* < 0.001 vs. control or NC group; ^#^*P* < 0.05, ^##^*P* < 0.01, and ^###^*P* < 0.001 vs. erastin+NC group; ^&^*P* < 0.05 and ^&&^*P* < 0.01 vs. erastin group.

**Figure 3:** Effects of REST on viability, ROS, ferroptosis, and neuron injury in erastin-induced LUHMES. After erastin stimulation, LUHMES were transfected with REST-overexpressed plasmid or sh-REST. (a) The levels of REST were evaluated through qRT-PCR analysis. (b) CCK-8 analyzed the impact of REST on the viability of cells. (c and d) Flow cytometry analyzed the impact of REST on ROS activity in the treated LUHMES cells. (e) TEM shows mitochondrial morphology. Scale bar = 2 *μ*m. Mitochondria are marked with blue arrows. (f) Western blotting analysis of REST, TH, NSE, ACSL4, and GPX4, and quantitative analysis of these proteins based on the western blotting results. Results were representative data from triplicate experiments, and data are means ± SD. ^∗∗∗^*P* < 0.001 vs. control group; ^#^*P* < 0.05, ^##^*P* < 0.01, and ^###^*P* < 0.001 vs. erastin+vector group; ^&^*P* < 0.05, ^&&^*P* < 0.01, and ^&&&^*P* < 0.001 vs. erastin+sh-NC group.

**Figure 4:** REST attenuates the effect of miR-494-3p on viability, ROS, ferroptosis, and neuron injury in erastin-induced LUHMES cells. Erastin-stimulated LUHMES were cotransfected with miR-494-3p inhibitor and sh-REST or REST-overexpressed plasmid and miR-494-3p mimics, respectively. (a and b) qRT-PCR showing the levels of miR-494-3p (a) and REST (b). (c) Cell viability was measured through the CCK-8 assay. (d) A Flow cytometer verified the change in ROS activity. (e) TEM images showing changes in mitochondrial morphology. Scale bar = 2 *μ*m. Mitochondria are marked with blue arrows. (f and g) Immunofluorescence images showing ACSL4 (f) and TH (g) expressions. Magnification: 200×, scale bar = 100 *μ*m. (h) Western blotting analysis showing REST, TH, NSE, ACSL4, and GPX4 levels. Results were representative data from triplicate experiments, and data are means ± SD. ^∗^*P* < 0.05, ^∗∗^*P* < 0.01, and ^∗∗∗^*P* < 0.001 vs. inhibitor+sh-NC group; ^#^*P* < 0.05, ^##^*P* < 0.01, and ^###^*P* < 0.001 vs. mimics+vector group.

**Figure 5:** SP1 reverses the roles of REST on viability, ROS, ferroptosis, and neuron injury in erastin-induced LUHMES cells. Erastin-stimulated LUHMES cells were coprocessed with REST and SP1 overexpression plasmids or REST shRNAs (sh-REST) and mithramycin. (a and b) The corresponding kit and qRT-PCR assay confirmed the transcription factor activity and expression of SP1. (c) Verification of SP1 transcription factor activity in REST-overexpressed or -silenced LUHMES cells after erastin stimulation. (d) CCK-8 was used to examine the change in cell viability. (e) ROS level was determined by flow cytometry. (f) TEM images showing mitochondrial morphology. Scale bar = 2 *μ*m. Mitochondria are marked with blue arrows. (g and h) Immunofluorescence staining showing ACSL4 (g) and TH (h) expressions. Magnification: 200×, scale bar = 100 *μ*m. (i) Western blotting highlights the changes in SP1, TH, NSE, ACSL4, and GPX4 expressions. Results were representative data from triplicate experiments, and data are means ± SD. ^∗^*P* < 0.05, ^∗∗^*P* < 0.01, and ^∗∗∗^*P* < 0.001 vs. erastin+vector group; ^###^*P* < 0.001 vs. erastin+REST+vector group; ^&^*P* < 0.05, ^&&^*P* < 0.01, and ^&&&^*P* < 0.001 vs. erastin+sh-NC group; ^^^*P* < 0.05, ^^^^*P* < 0.01, and ^^^^^*P* < 0.001 vs. erastin+sh-REST group.

**Figure 6:** SP1 can target ACSL4. (a) The binding sites between SP1 and ACSL4. (b and c) A dual-luciferase reporter assay was utilized to confirm the regulatory relationship between SP1 and ACSL4. (d and e) The regulatory effect of SP1 on ACSL4 was verified using CHIP (d) and EMSA assays (e). Results were representative data from triplicate experiments, and data are means ± SD. ^∗∗∗^*P* < 0.001.

**Figure 7:** miR-494-3p aggravates pathological changes, upregulates ACSL4, and downregulates TH in the substantia nigra and corpus striatum of the MPTP-induced PD mouse model. PD mouse model was established through MPTP induction, and then, PD model mice were addressed with miR-494-3p antagomir, miR-494-3p agomir, or ferrostatin-1. (a and b) qRT-PCR was utilized to analyze miR-494-3p (a) and REST (b) levels. (c) H&E staining determined the pathological changes in the substantia nigra and corpus striatum in the MPTP-induced PD mouse model. Magnification: 400×, scale bar = 50 *μ*m. (d) ACSL4 expression was assessed using an immunofluorescence assay. Magnification: 200×, scale bar = 100 *μ*m. (e) TH expression was identified using an immunohistochemistry assay. Magnification: 400×, scale bar = 50 *μ*m. Results were representative data from triplicate experiments, and data are means ± SD. Each group contained eight mice. ^∗∗∗^*P* < 0.001 vs. sham group; ^##^*P* < 0.01 and ^###^*P* < 0.001 vs. MPTP+NC group; ^&&^*P* < 0.01 vs. MPTP group.

## Data Availability

The datasets are available from the corresponding author upon reasonable request.

## Abbreviations

CHIP: Chromatin immunoprecipitation
GPX4: Glutathione peroxidase 4
H&E: Hematoxylin and eosin
LUHMES: Lund human mesencephalic cells
miRNAs: MicroRNAs
MPTP: 1-Methyl-4-phenyl-1,2,3,6-tetrahydropyridine
NC: Negative control
NSE: Neuron-specific enolase
PD: Parkinson's disease
qRT-PCR: Quantitative real-time polymerase chain reaction
REST: Repressor element-1 silencing transcription factor
ROS: Reactive oxygen species
SP1: Specificity protein 1
TEM: Transmission electron microscope
TH: Tyrosine hydroxylase.

## Additional Points

*Highlights*. (i) miR-494-3p inhibition prevents erastin-induced ferroptosis and neuron injury. (ii) REST is a target gene of miR-494-3p. (iii) REST inhibits ferroptosis, neuron injury, and ROS in erastin-induced LUHMES cells. (iv) SP1 is a downstream regulatory gene of REST. (v) SP1 can target ACSL4. (vi) miR-494-3p/REST/SP1/ACSL4 axis in Parkinson's disease.

## Supplementary Materials

Supplementary Materials Detailed methods for other experiments.

## References

[1] Tysnes O. B., Storstein A. (2017). Epidemiology of Parkinson's disease. *Journal of Neural Transmission (Vienna)*.

[2] Rai S. N., Singh P. (2020). Advancement in the modelling and therapeutics of Parkinson's disease. *Journal of Chemical Neuroanatomy*.

[3] Rai S. N., Singh P., Varshney R. (2021). Promising drug targets and associated therapeutic interventions in Parkinson's disease. *Neural Regeneration Research*.

[4] Reich S. G., Savitt J. M. (2019). Parkinson's disease. *The Medical Clinics of North America*.

[5] Rai S. N., Chaturvedi V. K., Singh P., Singh B. K., Singh M. P. (2020). Mucuna pruriens in Parkinson's and in some other diseases: recent advancement and future prospective. *Biotech*.

[6] Lu J., Wu M., Yue Z. (2020). Autophagy and Parkinson's disease. *Advances in Experimental Medicine and Biology*.

[7] Rocha E. M., De Miranda B., Sanders L. H. (2018). Alpha-synuclein: pathology, mitochondrial dysfunction and neuroinflammation in Parkinson's disease. *Neurobiology of Disease*.

[8] Mochizuki H., Choong C. J., Baba K. (2020). Parkinson's disease and iron. *Journal of Neural Transmission (Vienna)*.

[9] Michel P. P., Hirsch E. C., Hunot S. (2016). Understanding dopaminergic cell death pathways in Parkinson disease. *Neuron*.

[10] Kim T., Vemuganti R. (2017). Mechanisms of Parkinson's disease-related proteins in mediating secondary brain damage after cerebral ischemia. *Journal of Cerebral Blood Flow and Metabolism*.

[11] Mou Y., Wang J., Wu J. (2019). Ferroptosis, a new form of cell death: opportunities and challenges in cancer. *Journal of Hematology & Oncology*.

[12] Hirschhorn T., Stockwell B. R. (2019). The development of the concept of ferroptosis. *Free Radical Biology & Medicine*.

[13] Zeng X., An H., Yu F. (2021). Benefits of iron chelators in the treatment of Parkinson's disease. *Neurochemical Research*.

[14] Guiney S. J., Adlard P. A., Bush A. I., Finkelstein D. I., Ayton S. (2017). Ferroptosis and cell death mechanisms in Parkinson's disease. *Neurochemistry International*.

[15] Mahoney-Sánchez L., Bouchaoui H., Ayton S., Devos D., Duce J. A., Devedjian J. C. (2021). Ferroptosis and its potential role in the physiopathology of Parkinson's disease. *Progress in Neurobiology*.

[16] Kalayinia S., Arjmand F., Maleki M., Malakootian M., Singh C. P. (2021). MicroRNAs: roles in cardiovascular development and disease. *Cardiovascular Pathology*.

[17] Akkoc Y., Gozuacik D. (2020). MicroRNAs as major regulators of the autophagy pathway. *Biochimica et Biophysica Acta (BBA) - Molecular Cell Research*.

[18] Saliminejad K., Khorram Khorshid H. R., Soleymani Fard S., Ghaffari S. H. (2019). An overview of microRNAs: biology, functions, therapeutics, and analysis methods. *Journal of Cellular Physiology*.

[19] Han D., Dong X., Zheng D., Nao J. (2020). MiR-124 and the underlying therapeutic promise of neurodegenerative disorders. *Frontiers in Pharmacology*.

[20] Juźwik C. A., Drake S. S., Zhang Y. (2019). MicroRNA dysregulation in neurodegenerative diseases: a systematic review. *Progress in Neurobiology*.

[21] Luo M., Wu L., Zhang K. (2018). miR-137 regulates ferroptosis by targeting glutamine transporter SLC1A5 in melanoma. *Cell Death and Differentiation*.

[22] Geng L., Zhang T., Liu W., Chen Y. (2018). miR-494-3p modulates the progression of in vitro and in vivo Parkinson's disease models by targeting SIRT3. *Neuroscience Letters*.

[23] Deng C., Zhu J., Yuan J., Xiang Y., Dai L. (2020). Pramipexole inhibits MPP(+)-induced neurotoxicity by miR-494-3p/BDNF. *Neurochemical Research*.

[24] Liu H., Zhang Y., Yuan J. (2021). Dendritic cell-derived exosomal miR-494-3p promotes angiogenesis following myocardial infarction. *International Journal of Molecular Medicine*.

[25] Faversani A., Amatori S., Augello C. (2017). miR-494-3p is a novel tumor driver of lung carcinogenesis. *Oncotarget*.

[26] Lin H., Huang Z. P., Liu J. (2018). MiR-494-3p promotes PI3K/AKT pathway hyperactivation and human hepatocellular carcinoma progression by targeting PTEN. *Scientific Reports*.

[27] Brüll M., Spreng A. S., Gutbier S. (2020). Incorporation of stem cell-derived astrocytes into neuronal organoids to allow neuro-glial interactions in toxicological studies. *ALTEX*.

[28] Yang Y., Luo M., Zhang K. (2020). Nedd4 ubiquitylates VDAC2/3 to suppress erastin-induced ferroptosis in melanoma. *Nature Communications*.

[29] Gutbier S., Kyriakou S., Schildknecht S. (2020). Design and evaluation of bi-functional iron chelators for protection of dopaminergic neurons from toxicants. *Archives of Toxicology*.

[30] Campolo M., Casili G., Biundo F. (2017). The neuroprotective effect of dimethyl fumarate in an MPTP-mouse model of Parkinson's disease: involvement of reactive oxygen species/nuclear factor-*κ*B/nuclear transcription factor related to NF-E2. *Antioxidants & Redox Signaling*.

[31] Li D., Yang H., Ma J., Luo S., Chen S., Gu Q. (2018). MicroRNA-30e regulates neuroinflammation in MPTP model of Parkinson's disease by targeting Nlrp3. *Human Cell*.

[32] Hu Y. B., Zhang Y. F., Wang H. (2019). miR-425 deficiency promotes necroptosis and dopaminergic neurodegeneration in Parkinson's disease. *Cell Death & Disease*.

[33] Don Van B., Gouel F., Jonneaux A. (2016). Ferroptosis, a newly characterized form of cell death in Parkinson's disease that is regulated by PKC. *Neurobiology of Disease*.

[34] Zhang P., Chen L., Zhao Q. (2020). Ferroptosis was more initial in cell death caused by iron overload and its underlying mechanism in Parkinson's disease. *Free Radical Biology & Medicine*.

[35] Stockwell B. R., Jiang X. (2020). The chemistry and biology of ferroptosis. *Cell Chemical Biology*.

[36] Tang D., Chen X., Kang R., Kroemer G. (2021). Ferroptosis: molecular mechanisms and health implications. *Cell Research*.

[37] Bruni A., Pepper A. R., Pawlick R. L. (2018). Ferroptosis-inducing agents compromise in vitro human islet viability and function. *Cell Death & Disease*.

[38] Doll S., Freitas F. P., Shah R. (2019). FSP1 is a glutathione-independent ferroptosis suppressor. *Nature*.

[39] Chen X., Li J., Kang R., Klionsky D. J., Tang D. (2021). Ferroptosis: machinery and regulation. *Autophagy*.

[40] Wu J. R., Tuo Q. Z., Lei P. (2018). Ferroptosis, a recent defined form of critical cell death in neurological disorders. *Journal of Molecular Neuroscience*.

[41] Zhao Y., Li Y., Zhang R., Wang F., Wang T., Jiao Y. (2020). The role of erastin in ferroptosis and its prospects in cancer therapy. *Oncotargets and Therapy*.

[42] Gouel F., Do van B., Chou M. L. (2017). The protective effect of human platelet lysate in models of neurodegenerative disease: involvement of the Akt and MEK pathways. *Journal of Tissue Engineering and Regenerative Medicine*.

[43] Gunnarsson L. G., Bodin L. (2017). Parkinson's disease and occupational exposures: a systematic literature review and meta-analyses. *Scandinavian Journal of Work, Environment & Health*.

[44] Lai F., Jiang R., Xie W. (2018). Intestinal pathology and gut microbiota alterations in a methyl-4-phenyl-1,2,3,6-tetrahydropyridine (MPTP) mouse model of Parkinson's disease. *Neurochemical Research*.

[45] Chia S. J., Tan E. K., Chao Y. X. (2020). Historical perspective: models of Parkinson's disease. *International Journal of Molecular Sciences*.

[46] Zhang Q. S., Heng Y., Mou Z., Huang J. Y., Yuan Y. H., Chen N. H. (2017). Reassessment of subacute MPTP-treated mice as animal model of Parkinson's disease. *Acta Pharmacologica Sinica*.

[47] Jayaprakash S., le L. T. M., Sander B., Golas M. M. (2021). Expression of the neural REST/NRSF-SIN3 transcriptional corepressor complex as a target for small-molecule inhibitors. *Molecular Biotechnology*.

[48] Zhao Y., Zhu M., Yu Y. (2017). Brain REST/NRSF is not only a silent repressor but also an active protector. *Molecular Neurobiology*.

[49] Kawamura M., Sato S., Matsumoto G. (2019). Loss of nuclear REST/NRSF in aged-dopaminergic neurons in Parkinson's disease patients. *Neuroscience Letters*.

[50] Pajarillo E., Rizor A., Son D. S., Aschner M., Lee E. (2020). The transcription factor REST up-regulates tyrosine hydroxylase and antiapoptotic genes and protects dopaminergic neurons against manganese toxicity. *The Journal of Biological Chemistry*.

[51] O'Connor L., Gilmour J., Bonifer C. (2016). The role of the ubiquitously expressed transcription factor Sp1 in tissue-specific transcriptional regulation and in disease. *The Yale Journal of Biology and Medicine*.

[52] Dai C., Chen X., Li J., Comish P., Kang R., Tang D. (2020). Transcription factors in ferroptotic cell death. *Cancer Gene Therapy*.

[53] Zhang Q., Hu Y., Hu J. E. (2021). Sp1-mediated upregulation of Prdx6 expression prevents podocyte injury in diabetic nephropathy via mitigation of oxidative stress and ferroptosis. *Life Sciences*.

[54] Cai L. J., Tu L., Li T. (2020). Up-regulation of microRNA-375 ameliorates the damage of dopaminergic neurons, reduces oxidative stress and inflammation in Parkinson's disease by inhibiting SP1. *Aging (Albany NY)*.

[55] Han Y. P., Liu Z. J., Bao H. H., Wang Q., Su L. L. (2022). miR-126-5p targets SP1 to inhibit the progression of Parkinson's disease. *European Neurology*.

[56] Wang R., Yang Y., Wang H., He Y., Li C. (2020). MiR-29c protects against inflammation and apoptosis in Parkinson's disease model in vivo and in vitro by targeting SP1. *Clinical and Experimental Pharmacology & Physiology*.

[57] Wang S., Wen Q., Xiong B., Zhang L., Yu X., Ouyang X. (2021). Long noncoding RNA NEAT1 knockdown ameliorates 1-methyl-4-phenylpyridine-induced cell injury through microRNA-519a-3p/SP1 axis in Parkinson disease. *World Neurosurgery*.

[58] Yao L., Dai X., Sun Y. (2018). Inhibition of transcription factor SP1 produces neuroprotective effects through decreasing MAO B activity in MPTP/MPP+ Parkinson's disease models. *Journal of Neuroscience Research*.

[59] Wang Y., Cao R., Yang W., Qi B. (2019). SP1-SYNE1-AS1-miR-525-5p feedback loop regulates Ang-II-induced cardiac hypertrophy. *Journal of Cellular Physiology*.

[60] Vellingiri B., Iyer M., Devi Subramaniam M. (2020). Understanding the role of the transcription factor Sp1 in ovarian cancer: from theory to practice. *International Journal of Molecular Sciences*.

[61] Kuwata H., Hara S. (2019). Role of acyl-CoA synthetase ACSL4 in arachidonic acid metabolism. *Prostaglandins & Other Lipid Mediators*.

[62] Doll S., Proneth B., Tyurina Y. Y. (2017). ACSL4 dictates ferroptosis sensitivity by shaping cellular lipid composition. *Nature Chemical Biology*.

[63] Cheng J., Fan Y. Q., Liu B. H., Zhou H., Wang J. M., Chen Q. X. (2020). ACSL4 suppresses glioma cells proliferation via activating ferroptosis. *Oncology Reports*.

[64] Ma L. L., Liang L., Zhou D., Wang S. W. (2021). Tumor suppressor miR-424-5p abrogates ferroptosis in ovarian cancer through targeting ACSL4. *Neoplasma*.

[65] Cui Y., Zhang Y., Zhao X. (2021). ACSL4 exacerbates ischemic stroke by promoting ferroptosis-induced brain injury and neuroinflammation. *Brain, Behavior, and Immunity*.

[66] Zhang H. L., Hu B. X., Li Z. L. (2022). PKC*β*II phosphorylates ACSL4 to amplify lipid peroxidation to induce ferroptosis. *Nature Cell Biology*.

[67] Li Y., Feng D., Wang Z. (2019). Ischemia-induced ACSL4 activation contributes to ferroptosis-mediated tissue injury in intestinal ischemia/reperfusion. *Cell Death and Differentiation*.

[68] Xu Y., Li X., Cheng Y., Yang M., Wang R. (2020). Inhibition of ACSL4 attenuates ferroptotic damage after pulmonary ischemia-reperfusion. *The FASEB Journal*.

